The article "Application of Carbon Fiber Cement-Based Composites in Improving Construction Durability" was retracted in 2023. Reasons: signs of a paper mill; suspected computer-generated content; unreliable results or conclusions; concerns about the data.

# Application of Carbon Fiber Cement-Based Composites in Improving Construction Durability

**DOI:** 10.1155/2022/2323534

**Published:** 2022-08-24

**Authors:** Xiaoming Xu

**Affiliations:** Institute of Construction Engineering Technology, Changzhou Vocational Institute of Engineering, Changzhou, Jiangsu 213164, China

## Abstract

In order to improve the durability of building construction, this study proposes a construction method based on carbon fiber and cement-based composites. Analyze the mechanical properties of carbon fiber cement-based composites, combined with experiments to further analyze its advantages in building construction, to achieve the purpose of building durability construction. The experimental results show that the elastic modulus of CFRC samples with a 0.6% carbon fiber volume percentage is the largest. When the content of carbon fiber increases within a certain range, the elastic modulus of CFRC samples will also increase. *Conclusion*. The application of carbon fiber cement-based composites in building construction can effectively improve the durability of buildings and further improve the quality of buildings.

## 1. Introduction

However, with the further development of science and technology, traditional cement-based materials can no longer meet the changing needs brought about by social development [1]. The concept of intelligent structural materials has been proposed, and many scholars at home and abroad have invested in research on the intelligent modification of cement-based materials. Generally speaking, the modification of traditional cement-based materials is mainly achieved by adding other components with special properties. Carbon fiber is a kind of special fiber made of organic fiber by carbonization at high temperature in inert gas. It has many characteristics, such as lightweight, high strength, excellent conductivity, and high elastic modulus. It is favored by researchers at home and abroad in many fields [2].

A carbon fiber cement-based composite is a kind of composite material made of cement-based material as the base material and adding carbon fiber or its modified material. Due to the excellent properties of carbon fiber itself, compared with ordinary cement-based composites under the same conditions, carbon fiber cement-based composites have more excellent physical properties, and their compressive strength, tensile strength, flexural strength, and impermeability have been significantly improved. The resistivity of ordinary cement-based materials is generally between 10 and 11 Ω·m, which is basically nonconductive. The addition of carbon fiber to cement-based materials can significantly improve the conductivity of cement-based materials, greatly reduce their resistivity, and become a conductive material. This makes carbon fiber cement-based composites not only a building structure-bearing material but also an intelligent structural material, which can be applied to other fields, such as nondestructive testing of large cement-based structures such as roads, bridges, buildings, and so on; electromagnetic shielding of large equipment and instruments such as laboratories and research institutes; and snow melting and ice melting in cold weather of roads and airports [3].

The quality and safety inspection of construction projects is an important measure to ensure the safety and reliability of construction projects. At present, the quality inspection of construction projects in China is mainly carried out through the safety and durability of building structures. The safety of the building structure is an important guarantee to ensure that the construction project will not have cracks, collapses, and other events, and the durability of the building structure determines the service life of the construction project.

Therefore, combined with the above, the application of carbon fiber cement-based composites in building construction can effectively improve the durability of buildings and ensure the safety and reliability of construction projects.

## 2. Literature Review

Cement is the building material with the largest output and used in today's construction projects. Since the advent of Portland cement, cement products and materials such as mortar, concrete, and reinforced concrete have been born. The average annual consumption of cement-based composites in China is about 10^8^ m^3^. Production and consumption are far more than in other countries in the world. It can be seen from this that cement materials will be the most important engineering construction materials in China for a long time until new materials that replace cement appear. However, the toughness of cement mortar material is relatively poor, and it is not suitable for use in structures with high tensile and bending requirements, so it is impossible to complete the mechanical design requirements of long-span structures alone. Later, the emergence of reinforced concrete structures solved the defect of cement materials, in which steel bars could bear strong tension and concrete could bear strong pressure. The combination of the two can give full play to their respective advantages, thus effectively overcoming the defects of poor tensile performance and limited scope of application of cement mortar materials [4]. Adding steel bars to concrete greatly enhances the tensile strength and flexural strength of concrete and further expands the application range of cement mortar materials. However, the reinforcement is not corrosion-resistant. Reinforced concrete structures also have their own shortcomings. In order to overcome this shortcoming, we must find new materials.

Adding a small amount of chopped fiber to the mixing process of cement mortar materials is an effective method to enhance the tensile and compressive properties of cement mortar. The addition of chopped fiber can enhance the tensile strength, crack strength, and fatigue strength of cement mortar materials, so that they have excellent mechanical properties. Various chopped fibers are added into cement mortar materials to enhance the mechanical properties of cement-based materials. This method of adding chopped fibers has a long history of development [5]. The types of added fibers can range from early crops such as wheat straw and hemp, and later fibers made of asbestos to glass fibers and steel fibers are now used. These reinforcing fibers can improve the performance of cement and can also be widely used in actual buildings. The use of asbestos and glass fiber in cement materials is a monument in the history of architecture. Later, steel fiber came into being with the development of fiber materials. The excellent performance of steel fiber makes it widely used in strengthening the mechanical properties of cement mortar materials. However, most fibers have their own inevitable shortcomings [6]. For example, fibers made of asbestos are carcinogenic, and fibers made of glass and steel are easy to corrode under the strong alkali conditions of cement mortar and lose their role in cement mortar materials [7]. Compared with the previous fibers, carbon fiber is nontoxic and harmless and has good stability in cement mortar, so it is more suitable to be used as reinforcement in cement mortar. Carbon fiber has been developed rapidly because of its many advantages, especially in cement-based composites.

A carbon fiber cement-based composite is a combination of a certain amount of chopped carbon fiber and cement material, which is called CFRC for short. CFRC has many superior properties to cement mortar materials. For example, the toughness and tensile strength of CFRC are better than those of cement mortar materials. Its addition can also reduce the dry shrinkage of cement mortar materials. In addition to its advantages in mechanical properties, CFRC also has special functions in temperature sensitivity, electric heating, pressure-sensitive, electromagnetic shielding, and other aspects [8]. In winter, when encountering rain and snow, the road surface is often covered with ice and snow. Vehicles driving on this kind of road are prone to traffic accidents. Highways are often closed because the road surface is covered with ice and snow, so it is necessary to find effective ways to solve this problem. The efficiency of ordinary snow and ice removal methods is low. When CFRC is used as a pavement material, using the conductivity of CFRC and the power on and heating function of conductive materials can play a role in snow and ice removal, so as to effectively solve this problem; CFRC is sensitive to compressive stress. Applying pressure to the CFRC sample can change the resistivity of the sample. Using this characteristic, we can master the stress and strain of CFRC at any time by monitoring the change of CFRC resistivity at any time. Using this special performance of CFRC, we can also monitor the damage to a building structure and provide a guarantee for its safety, so as to achieve the role of the sensor; some special building structures have high-temperature requirements. By using the characteristic that CFRC is very sensitive to temperature changes, the function of automatically adjusting its temperature can be achieved; using the relationship between CFRC load and resistance, the load of the structure can be known through the current, so as to play its load-bearing role on the vehicle; many electromagnetic waves are harmful to the human body. Using the electromagnetic shielding performance of CFRC can make people's living environment free from the interference of harmful electromagnetic fields and achieve the purpose of protecting human health. All these show that carbon fiber cement-based composites have a wide range of applications. Its application can bring many benefits to life, so its application scenario is also very broad, and its research is more and more practical value [9].

Based on the above research, this study proposes to apply carbon fiber cement-based composites to construction, and through the experiment and analysis of their mechanical properties, to evaluate the durability of this material in the construction industry, so as to ensure durability in construction and ensure construction safety.

## 3. Research Methods

### 3.1. Analysis of Mechanical Properties by the Differential Method and Variational Method

The differential equivalent medium for calculating the mechanical properties of composites by the differential method was first found. Later, this definition is used to calculate the elastic modulus of composite materials. What it builds is a process in which inclusions are gradually added to the matrix material. First, a small amount of inclusions are added to the matrix material to homogenize the whole material. Then add the inclusion material, homogenize it, repeat the project continuously, and finally obtain the mechanical properties of the composite with a certain volume content of inclusions [10]. The cyclic steps of adding and homogenizing by the differential method are shown in Figure 1.

The variational method is to solve the mechanical properties of composite materials by using the variational principle. This method is obviously different from the above methods. Through the variational method, the range of some mechanical property parameters of composites is derived.

CFRC is a new material composed of carbon fiber and cement base. Chopped carbon fiber and cement base exist in an independent form in the whole structure. On the surface, this material belongs to composite materials. To study the mechanical properties of CFRC, we can start with the mechanical research method of composite materials. At present, most of the research methods on the mechanical properties of CFRC are based on the first research method, that is, the macro method based on experiments [11]. There is little research on the mechanical properties of CFRC from the mesoscopic point of view. Moreover, when using the macro method, the experiment has certain requirements for the manufacturing process and curing of CFRC samples. As long as there is a certain deviation in these aspects, the experimental results will be different. Therefore, the analysis of CFRC mechanical problems must combine the two methods described above, verify, and complement each other. In this way, the mechanical properties of CFRC can be effectively discussed. In this study, the mechanical properties of CFRC are obtained by the theoretical method and then compared with the experimental results to see whether the meso method is suitable for calculating the mechanical properties of CFRC [12].

Under the electron microscope, the broken section of CFRC can clearly see that the distribution of carbon fiber in cement mortar is random and irregular. In order to study the mechanical properties of CFRC by using the mesostructural mechanics method of composite materials, it is necessary to homogenize the CFRC structure first. Assuming that the carbon fibers are evenly distributed in the cement base, the homogenized CFRC can be regarded as a statistical uniform field, and then, the mechanical problems of CFRC can be solved by using the mesostructural mechanics method of composite materials. On this basis, the mechanical problems of CFRC can be solved by using the mesomechanical method [13].

### 3.2. Theoretical Analysis of CFRC Mechanical Properties

#### 3.2.1. Representative Units and Statistically Uniform Materials

General composite materials, such as CFRC, are composed of different component materials. By observing the fracture section of CFRC samples under the electron microscope, we can clearly see the distribution of carbon fibers in the cement base. In CFRC, concrete is a continuous matrix material, and carbon fibers are dispersed in the matrix material [14]. Therefore, the mesostructure of CFRC is very complex, the distribution of carbon fibers is random, and its length is inconsistent. Therefore, it is difficult to describe the mesostructure of CFRC with mathematical models or formulas.

When considering the overall mechanical properties of CFRC, its mesostructure is often simplified. First, it will be assumed that all reinforcing phases (carbon fibers) have the same shape and size. For example, in CFRC, it can be assumed that the length of fiber is the same and the diameter of the fiber is also the same. Second, assuming that the fibers are completely uniformly distributed in the matrix material, the mesostructure of CFRC has periodicity and uniformity [15]. After homogenization, CFRC is composed of many cells. The unit cell can also be regarded as the meso-representative unit of CFRC, which can represent the mechanical properties of CFRC.

The homogenized CFRC can also be regarded as a statistically homogeneous material. When the uniform stress or strain defined by the uniform boundary condition is applied to the statistically uniform material, the stress-strain field in the material can be considered as a uniform statistical field, and the field variables of the mesoelement of the material are calculated, that is, the mechanical properties of the homogenized CFRC are obtained [15].

#### 3.2.2. Uniform Boundary Conditions

In order to form the statistical uniform field of CFRC, it is necessary to impose a uniform boundary condition on the assumed completely uniform CFRC. There are mainly two kinds of uniform boundary conditions, which are expressed as follows:

(1) Uniform stress boundary conditions:
  (1) $$\begin{array}{c} u_{i}^{0}\left(S\right)=\varepsilon_{ij}^{0}x_{i}. \end{array}$$
Where S is the statistical uniform material boundary, *u*_*i*_^0^(*S*) is the applied boundary displacement, *ε*_*ij*_^0^ is the constant strain, *x*_*i*_ is the axial coordinate, and *i*, *j* = 1, 2, 3.
(2) Uniform strain boundary condition:
  (2) $$\begin{array}{c} T_{i}\left(S\right)=\sigma_{ij}^{0}n_{j}. \end{array}$$
Where *T*_*i*_(*S*) is the boundary load, *σ*_*ij*_^0^ is the constant strain, and *n*_*j*_ is the outer discovery direction of the boundary.

In the homogenized CFRC, the statistical uniform field variable of the material is the same as the volume average field variable of the material. Therefore, in the elastic field, the statistical uniform value of the representative element of CFRC can be expressed by the volume average value of the representative element.

The average strain of statistical uniform material CFRC:

(3) $$\begin{array}{c} \bar{\varepsilon_{ij}}=\frac{1}{V}{∭}_{V}\varepsilon_{ij}dv. \end{array}$$

Average stress of statistical uniform material CFRC:

(4) $$\begin{array}{c} \bar{\sigma_{ij}}=\frac{1}{V}{∭}_{V}\sigma_{ij}dv. \end{array}$$

### 3.3. Experimental Study on Mechanical Properties of FRC

The main purpose of this experiment is to measure the stress-strain relationship of CFRC samples with different carbon fiber volume percentages and obtain the actual mechanical property parameters of CFRC materials, so as to further test the correctness of the theoretical research results [16].

#### 3.3.1. Raw Materials

This study presents a retrospective analysis of the experimental materials selected for mechanical properties:

  Material 1: cement: the cement model used in the experiment is 42.5.
  Material 2: fine sand: natural river sand, repeatedly filtered with a sieve, is fine gravel.
  Material 3: PAN-based carbon fiber: its mechanical property parameters are shown in Table 1.
  Material 4: dispersant: methylcellulose. The main function is to separate the carbon fiber and finally achieve the purpose of a uniform distribution of carbon fiber in the cement base.
  Material 5: water reducer: the main function are to disperse cement, reduce the amount of water in the mixing process, and improve the strength of concrete samples.

#### 3.3.2. Equipment and Instruments Used in the Experiment

This study presents a retrospective analysis of the instruments used in the experiment on the mechanical properties of carbon fibers.

1. Cement paste mixer is mainly used to mix concrete mortar and carbon fiber so that carbon fiber is evenly distributed in concrete mortar
2. Cement mortar vibrating table, main purpose: when making CFRC samples, make the samples vibrate and form, so as to prevent the existence of cavities in the samples
3. Tray balance is mainly used for weighing the mass of sand, cement, and water
4. JA series electronic balance is mainly used for raw materials with high weighing accuracies, such as carbon fiber; quality of water reducing agent, and dispersant.
5. Electrohydraulic servo universal testing machine. Main use: when the CFRC sample is under pressure, measure the relationship between the stress and strain of the sample, and measure the mechanical property parameters of the material [17].

#### 3.3.3. Experimental Process

In this study, the experimental process of mechanical properties analysis of carbon fiber is analyzed retrospectively.

*(1) Sample Raw Material Ratio.* The principle of selecting the mix proportion: first, the mix proportion of cement mortar is selected. The mix proportion of cement mortar selected in this experiment is the proportion of cement, sand, and water according to the mass ratio of 1 : 1 : 0.3. Change the parameters of carbon fiber and the dosage of water and dispersant appropriately under the condition that the cement and sand remain unchanged, so as to ensure the appropriate performance of CFRC samples.

Through calculation, when the volume percentage of carbon fiber in CFRC is 0.3%, the mass ratio of each component's raw material is shown in Table 2.

When the volume percentage of carbon fiber in CFRC is 0.6%, the mass ratio of each component's raw material is shown in Table 3.

When the volume percentage of carbon fiber in CFRC is 0.9%, the mass ratio of each component's raw material is shown in Table 4.

*(2) CFRC Sample Making and Experimental Test*. In this study, the fabrication and experimental testing of CFRC samples are analyzed retrospectively.

1. Prepare the principle of each component according to different mass proportions
2. Take a container, pour water into the container, add dispersant to the water, stir the dispersant and water, and make the dispersant fully dissolved in the water
3. Add the carbon fiber into the vessel containing dispersant and water, stir by hand to separate the carbon fiber, then add other materials prepared in front, pour them into the cement paste mixer, stir for a period of time, and then take out the cement base containing carbon fiber
4. Slowly pour the mixed carbon fiber mortar into the mold, place the mold on the shaking table, and vibrate for 15 minutes to make it dense. In this way, a 100*∗*100*∗*100 mm^3^ CFRC sample is made. Demould after 24 hours under normal temperature and maintain in the curing box for one month [18].
5. On the electrohydraulic servo universal testing machine, apply pressure to the sample at the loading speed of 1 kn/s

## 4. Experimental Results and Analysis

Through the compression loading experiment of the electrohydraulic servo universal testing machine, the compression load and compression displacement diagrams of CFRC samples with different carbon fiber volume percentages are obtained on the associated computer. The points with the same displacement are taken in each diagram, and the data for each point are processed according to the actual situation [19]. The compressive stress of the sample is obtained by dividing the compressive load of each point after treatment by the surface area of the sample, and the compressive strain is obtained by dividing the compressive displacement by the size of the sample. Finally, the stress-strain relationship of CFRC samples with three carbon fiber volume contents is obtained, as shown in Figure 2.

By observing the stress-strain relationship of CFRC samples in Figure 2, it is found that the elastic modulus of CFRC samples with a volume percentage of carbon fiber of 0.6% is the largest, and it can be concluded that when the content of carbon fiber increases within a certain range, the elastic modulus of CFRC samples will also increase [20]. When observing the cross-sections of CFRC samples with different carbon fiber contents with an electron microscope, it can be clearly seen that when the carbon fiber content is relatively high. Therefore, the mechanical properties of CFRC specimens will decrease with the increase of carbon fiber content.

## 5. Conclusion

In this study, a carbon fiber cement composite material is proposed and its mechanical properties are analyzed in order to put it into construction and improve the durability of construction. The experimental results show that the elastic modulus of CFRC samples with a 0.6% carbon fiber volume percentage is the largest. When the content of carbon fiber increases in a certain range, the elastic modulus of CFRC samples will also increase. It can be seen that carbon fiber cement composite has strong mechanical properties, and its application to building construction can greatly improve the durability of construction.

## Figures and Tables

**Figure 1:** Differential equivalence principle.

**Figure 2:** Stress-strain diagram of CFRC sample.

**Table 1:** Mechanical property parameters of carbon fiber.

Diameter/*μ*m	Tensile strength/GPa	Modulus of elasticity/GPa	Poisson's ratio	Elongation/%
6.5	4.0	240	0.26	1.4

**Table 2:** Mass ratio of CFRC materials.

Sand/cement (%)	Water/cement (%)	Carbon fiber/cement (%)	Water reducer/cement (%)	Dispersant/cement (%)
100	30	0.5	15	0.5

**Table 3:** Mass ratio of CFRC materials.

Sand/cement (%)	Water/cement (%)	Carbon fiber/cement (%)	Water reducer/cement (%)	Dispersant/cement (%)
100	32	1	0.5	1

**Table 4:** Mass ratio of CFRC materials.

Sand/cement (%)	Water/cement (%)	Carbon fiber/cement (%)	Water reducer/cement (%)	Dispersant/cement (%)
100	34	1.5	0.5	1.5

## Data Availability

The data used to support the findings of this study are available from the corresponding author upon request.

## References

[1] Zhang W., Hou D., Ma H. (2021). Multi-scale study water and ions transport in the cement-based materials:from molecular dynamics to random walk. *Microporous and Mesoporous Materials*.

[2] Yang F. (2022). Cycling-induced structural damage/degradation of electrode materials–microscopic viewpoint. *Nanotechnology*.

[3] Lin J., Wu J., Fan E. (2022). Environmental and economic assessment of structural repair technologies for spent lithium-ion battery cathode materials. *International Journal of Minerals, Metallurgy and Materials*.

[4] Jean-St-Laurent M., Dano M. L., Potvin M. J. (2022). Effect of extreme cold temperatures on quasi-static indentation and impact behavior of woven carbon fiber epoxy composite sandwich panels with nomex honeycomb core. *Journal of Sandwich Structures and Materials*.

[5] Chen J., Li Z., Fu Z. (2021). A comparative analysis of carbon fiber–reinforced polymers subjected to lightning damage tests with conical electrodes and jet diverting electrodes. *Journal of Testing and Evaluation*.

[6] Zhu H., Zhou H., Gou H. (2021). Evaluation of carbon fiber dispersion in cement-based materials using mechanical properties, conductivity, mass variation coefficient, and microstructure. *Construction and Building Materials*.

[7] Xu W., Jalal M., Zakira U., Wang L. (2021). Study on the mechanical properties and durability of carbon fiber reinforced lime-based mortar. *IOP Conference Series: Earth and Environmental Science*.

[8] Hongling L., Yude D., Lei Q., Juxin S. (2022). Belt width optimization for tire durability enhancement. *Proceedings of the Institution of Mechanical Engineers - Part D: Journal of Automobile Engineering*.

[9] Shunmugasundaram M., Praveen Kumar A., Ahmed Ali Baig M., Kasu Y. (2021). Investigation on the effect of nano fillers on tensile property of neem fiber composite fabricated by vacuum infused molding technique. *IOP Conference Series: Materials Science and Engineering*.

[10] Sun K. C., Noh J. W., Choi Y. O., Jeong S. H., Kim Y. S. (2021). Zeolite and short-cut fiber-based wet-laid filter media for particles and heavy metal ion removal of wastewater. *Journal of Industrial Textiles*.

[11] Rosol T. J., Witorsch R. J. (2021). Ethyl acrylate (ea) exposure and thyroid carcinogenicity in rats and mice with relevance to human health. *Regulatory Toxicology and Pharmacology*.

[12] Cui C., Wang L., Liu W., Xu S., Liu X. (2021). Study on emission characteristics and health effects of volatile organic compounds in child seats. *IOP Conference Series: Earth and Environmental Science*.

[13] Zhang J., Wang X., Fu X. (2021). High mechanic enhancement of chopped carbon fiber reinforced-low-density unsaturated polyester resin composite at low preparation temperature with facile polymerization. *Materials*.

[14] Kornilitsina E. V., Lebedeva E. A., Astaf’Eva S. A., Trukhinov D. K. (2021). Modification of carbon fiber by magnetite particles. *IOP Conference Series: Materials Science and Engineering*.

[15] Bakamal A., Ansari R., Hassanzadeh-Aghdam M. K. (2021). Bending, free vibration, and buckling responses of chopped carbon fiber/graphene nanoplatelet-reinforced polymer hybrid composite plates: an inclusive microstructural assessment. *Proceedings of the Institution of Mechanical Engineers—Part C: Journal of Mechanical Engineering Science*.

[16] Huang R., Yang X. (2022). Analysis and research hotspots of ceramic materials in textile application. *Journal of Ceramic Processing Research*.

[17] Jayakumar J., Nagaraj B., Chacko S., Ajay P. (2021). Conceptual implementation of artificial intelligent based E-mobility controller in smart city environment. *Wireless Communications and Mobile Computing*.

[18] Zhao X., Liu X., Liu J., Chen J., Fu S., Zhong F. (2019). The effect of ionization energy and hydrogen weight fraction on the non-thermal plasma volatile organic compounds removal efficiency. *Journal of Physics D: Applied Physics*.

[19] Huang Z., Li S. (2022). Reactivation of learned reward association reduces retroactive interference from new reward learning. *Journal of Experimental Psychology: Learning, Memory, and Cognition*.

[20] Zhang Q. (2021). Relay vibration protection simulation experimental platform based on signal reconstruction of MATLAB software. *Nonlinear Engineering*.

